# *Lactobacillus pentosus* Alleviates Lipopolysaccharide-Induced Neuronal Pyroptosis via Promoting BIRC3-Mediated Inactivation of NLRC4

**DOI:** 10.1155/2022/2124876

**Published:** 2022-06-23

**Authors:** Ming Hu, Zhongying Shao

**Affiliations:** ^1^Department of Neurology, The Second Affiliated Hospital of Shandong First Medical University, Tai'an 271000, Shandong, China; ^2^Department of Liver Diseases, Tai'an Traditional Chinese Medicine Hospital, Tai'an 271000, Shandong, China

## Abstract

**Objective:**

Neurodegenerative disease is a common neurodegenerative disorder. *Lactobacillus pentosus* (*L. pentosus*) plays a neuron-protective role. This study aimed to investigate the effects of *L. pentosus* on neurodegenerative diseases.

**Methods:**

Cells were treated with lipopolysaccharide (LPS) to establish neurodegenerative diseases model in vivo and with *L. pentosus* strain S-PT84. Reverse transcription-quantitative PCR (RT-qPCR) was applied to determine mRNA levels. Western blot was performed to detect protein expression. Cellular behaviors were detected using Cell Counting Kit-8 (CCK-8), flow cytometry, and TdT-mediated dUTP nick-end labeling (TUNEL) assay. The interaction between baculoviral IAP repeat containing 3 (BIRC3) and NLR family CARD domain containing 4 (NLRC4) was predicted by STING and verified by western blot.

**Result:**

*L. pentosus* suppressed LPS-induced pyroptosis and promoted the cell viability of neurons. Additionally, *L. pentosus* suppressed the release of proinflammatory cytokines (interleukin 1 beta (IL-1*β*) and IL-18) and the protein expression of pyroptosis biomarkers (cleaved caspase1 (CL-CASP1) and N-terminal fragment gasdermin *D* (GSDMD-N)). Moreover, *L. pentosus* upregulated BIRC3, which induced the inactivation of NLRC4. However, BIRC3 knockdown alleviated the effects of *L. pentosus* and induced neuronal degeneration.

**Conclusion:**

*L. pentosus* may play a neuron-protective role via regulating BIRC3/NLRC4 signaling pathways. Therefore, *L. pentosus* may be a promising strategy for neurodegenerative diseases.

## 1. Introduction

Dementia is a common neurodegenerative disease, characterized by progressive cognitive degeneration, which induces huge burden on public health [1]. Elder neuron degeneration is the main cause of dementia [2]. Recently, Marchetti reveals that the changes in microenvironment, including inflammation, are a key factor for neural degeneration [3]. Hence, to develop a new strategy for suppressing inflammation-induced neurodegeneration is in urgent need.

Pyroptosis is a form of programmed cell death executed by Gasdermin D (GSDMD) [4] The activation of inflammasomes, such as NLR family pyrin domain containing 1 (NLRP1) [5], NLR family CARD domain containing 4 (NLRC4), NLRP3, NLRP6, and NLRP12 [6, 7], cleave caspase1 (CASP1) (canonical pathway) or CASP11 (noncanonical pathway), which promotes the N-terminal fragment GSDMD (GSDMD-N) assembling into cell membrane. The accumulation of GSDMD-N induces pore formation, the release of IL-1*β* and IL-18, and cell death [8, 9]. Previous studies evidence that the pyroptosis of neurons induces pathogenesis of optic nerve disorders and cerebral ischemia as well as Alzheimer's disease [10–12]. However, the molecular mechanisms underlying neuron pyroptosis have not been fully elucidated.

Probiotics are considered to be a safe alternative therapy for many diseases, including cancer and neural disorders [13, 14]. According to the Food and Drug administration (FDA), moderate-taken probiotics bring healthy benefits to the host [15]. Generally, probiotics can actively change the host's intestinal microbiota and improve health. *Lactobacillus pentosus* (*L. pentosus*), a member of probiotics from intestinal flora, plays a neuron-protective role and mitigates aging- and scopolamine-induced memory impairment [16, 17]. However, probiotic-based treatments for memory loss, especially for patients with neurodegenerative diseases, and their clinical outcomes are not fully documented.

Baculoviral IAP repeat containing 3 (BIRC3) is a member of inhibitor of apoptosis proteins (IAPs) [18]. BIRC3 suppresses cell apoptosis via inactivating CASPs cascades [19]. The abnormal levels of BIRC3 are closely associated with tumorgenesis [20, 21], inflammatory response [22], and immune disorders [23]. For instance, the activation of BIRC3 induces chemoresistance of colorectal cancer [24]. BIRC3 modulates canonical nuclear factor kappa B (NF-*κ*B) target gene activation to attenuate inflammation, which promotes the development of splenic marginal zone lymphoma [25]. Moreover, BIRC3 promotes the cell survival of neurons [26]. However, the roles of BIRC3 in neurodegenerative diseases are still unclear. This study investigated the potentials of BIRC3. BIRC3 protected against neuronal degeneration via suppressing inflammation-induced pyroptosis.

## 2. Materials and Methods

### 2.1. Cell Culture

Human neuroblastoma cell lines SH-SY5Y were provided by American type culture collection (ATCC), USA. Cells were cultured in Dulbecco's modified Eagle's medium (DMEM) medium containing 10% FBS and 1% penicillin/streptomycin at 37°C with 5% CO_2_.

Cells (2 × 10^5^ cells) were incubated with 10 *μ*g/L of lipopolysaccharide (LPS) and/or *L. pentosus* strain S-PT84 (*L. pentosus*, 5 × 10^7^ cells/ml, Synbiotech Inc., Kaohsiung, China).

### 2.2. Cell Transfection

Sh-BIRC3 and its negative control were provided by GenePharm, Shanghai. Cells were transfected using Lipofectamine® 3000 for 48 h. After transfection, cells were used in the following experiments.

### 2.3. Reverse Transcription-Quantitative PCR (RT-qPCR)

Total RNA was collected from SH-SY5Y cells. RNA was reversely transcribed into cDNA using a reverse transcription kit (Applied Biosystems, USA). Then, PCR was performed using SYBR Premix Ex Taq (Takara, Japan). GAPDH served as loading control. Relative mRNA levels were calculated using the 2^−ΔΔCq^ method. Each independent experiment was conducted in triplicate.

### 2.4. Western Blot

Total protein was extracted from SH-SY5Y cells. Protein concentration was measured using a bicinchonininc acid (BCA) kit. The protein was separated using 12% SDS-PAGE. Afterwards, the separated protein was moved onto polyvinylidene difluoride (PVDF) membranes, which was then sealed by 5% skimmed milk. The membranes were incubated with primary antibodies against IL-1*β*, IL-18, procaspase1, cleaved caspase1, GSDMD-N, BIRC3, NLRP3, NLRC1, NLRP3, NLRC4, and glyceraldehyde-3-phosphate dehydrogenase (GAPDH) at 4°C overnight. Next day, the membranes were incubated with secondary antibodies. GAPDH was used as the loading control. Subsequently, the bands were captured using an efficient chemiluminescence (ECL) kit and analyzed using the ImageJ software.

### 2.5. Coimmunoprecipitation (Co-IP)

Cells were collected and lysed. Then, cell lysates were centrifuged at 12,000 × g and immunoprecipitated with specific antibodies. Afterwards, the proteins were coprecipitated and isolated using 12% SDS-PAGE. Immunoblotting was analyzed with antianalysis with the indicated primary antibodies against BIRC3, NLRC4, and GAPDH.

### 2.6. Cell Viability

Cells were seeded into 24-well plates (2 × 10^3^ cells/well). After incubated with *L. pentosus* for 48 h, cells were cultured with Cell Counting Kit-8 (CCK-8) regents for 4 h. Subsequently, optic density was determined using a microplate at 450 nm.

### 2.7. Flow Cytometry

Cell pyroptosis was determined using an FAM-FLICA Caspase-1 Assay Kit. Cells were seeded in 6-well plates. After centrifugation at 1200 × g for 15 min, the supernatants were collected. Then, the cells were stained cultured with propidium iodide (PI). Subsequently, a flow cytometry was used to calculate the pyroptosis rates: active caspase1 + PI double positive cells/total cells × 100%.

### 2.8. TdT-Mediated dUTP Nick-End Labeling (TUNEL) Assay

Cells were collected and fixed with 4% paraformaldehyde. After washed with 5% PBS, cells were cultured with TUNEL solutions. Then, the cells were counterstained with DAPI. Finally, TUNEL positive cells were captured using a fluorescence microscope.

### 2.9. Statistical Analysis

All data were evaluated using GraphPad 6.0. and represented as mean ± SD. The comparison was performed using Student's *t*-test and one-way ANOVA. *P* < 0.05 dictated significant difference.

## 3. Results

### 3.1. The Cell Viability of Neuron Cells

To investigate the effects of *Lactobacillus pentosus* (*L. pentosus*) on neuronal degeneration, cells were cultured with *L. pentosus*. As shown in Figure 1, there were no significant changes in the cell viability of SH-SY5Y cells.

### 3.2. *L. pentosus* Suppresses Inflammatory Response in SH-SY5Y Cells

Inflammation is a key factor for neuronal degeneration. To verify the effects of *L. pentosus*, SH-SY5Y cells were exposed to LPS. As shown in Figures 2(a)–2(c), LPS significantly increased the release of IL-1*β* and IL-18, which was antagonized by *L. pentosus*. These results were consistent with that from western blot. *L. pentosus* treatment markedly alleviated the effects of LPS and suppressed the protein expression of IL-1*β* and IL-18.

### 3.3. *L. pentosus* Inhibits the Pyroptosis of SH-SY5Y Cells

Cellular functions were detected using flow cytometry and TUNEL assay. As shown in Figure 3(a), *L. pentosus* significantly decreased PI and active caspase1-positive cells induced by LPS. Additionally, LPS-mediated increase in TUNEL-positive cells was abated by *L. pentosus* treatment (Figure 3(b)). To further verify the effects of *L. pentosus* on LPS-induced neuronal cell death, we determined the protein expression of pyroptosis biomarkers. LPS exposure significantly increased the protein expression of cleaved caspase1 and GSDMD-N (Figure 3(c)), which was alleviated by *L. pentosus*.

### 3.4. *L. pentosus* Increased the Expression of BIRC3

Previous studies report that BIRC3 plays a neuron-protective role. We then determined the expression of BIRC3 in neurons. As shown in Figure 4(a), the mRNA expression of BIRC3 was significantly decreased in the LPS group; however, *L. pentosus* treatment significantly increased BIRC3 mRNA levels compared with the LPS group (Figure 4(a)). Moreover, *L. pentosus* also increased the protein expression of BIRC3 (Figure 4(b)).

### 3.5. BIRC3 Knockdown Induces the Release of Proinflammatory Cytokines

The rescue assay was performed to verify the roles of BIRC3 in neuronal degeneration. As shown in Figure 5(a), sh-BIRC3 significantly suppressed the mRNA and protein expression of BIRC3 compared with LPS + *L. pentosus* + sh-NC group. BIRC3 knockdown significantly suppressed the cell viability of SH-SY5Y cells (Figure 5(c)). Additionally, BIRC3 markedly promoted the release and protein expression of proinflammatory cytokines, such as IL-1*β* and IL-18 (Figures 5(d) and 5(e)).

### 3.6. BIRC3 Knockdown Induced the Pyroptosis of SH-SY5Y Cells

As shown in Figures 6(a) and 6(b), downregulated BIRC3 significantly increased the PI + active caspase1-positive cells as well as TUNEL-positive cells. Moreover, BIRC3 knockdown significantly increased the protein expression of cleaved caspase1 and GSDMD-N (Figure 6(c)).

### 3.7. BIRC3 Inactivates NLRC4 Inflammasome

We further investigated the underlying molecular mechanisms that BIRC3 inhibited neuronal pyroptosis. The online database STING showed that the potential genes interacts with BIRC3 (Figure 7(a)). The results showed that BIRC3 could interact with NLRC4; however, the expression of NLRP1, NLRP3, NLRP4, and NLRP1 showed no significant changes after transfection with sh-BIRC3.

## 4. Discussion

In this study, *L. pentosus* play a neuron-protective role. *L. pentosus* suppressed inflammatory response and pyroptosis of neuron cells. Moreover, *L. pentosus* upregulated BIRC3, suppressing the inactivation of NLRC4 inflammasome. Hence, *L. pentosus* may be a promising therapy for neurodegenerative diseases.

The activation of inflammasomes increases cytotoxicity and contributes to the pyroptosis of neurons, which is a key factor for memory loss and cognitive impairment [27]. For instance, the activation of NLRC4 inflammasome interacts with CASP1, IL-1*β*, and p-Tau to contribute to neuroinflammation and memory impairment [28]. High levels of caspase1 induces human mild cognitive impairment and brain functions in patients with Alzheimer's disease, while depletion of NLRP3 promotes spatial memory and suppresses M2 polarization of microglia and deposition of amyloid-*β* [29]. NLRP1 deficiency suppresses the pyroptosis of neurons and improves cognitive capability [30]. These results suggested that inactivation of inflammasomes may be an effective strategy for neurodegenerative diseases. In this study, LPS exposure upregulated NLRC4 in neurons. The activation of NLRC4 inflammasome cleaved CASP1 and induced pore formation [31], which further contributed to neuronal pyroptosis. However, *L. pentosus* treatment restored neuronal cellular functions, manifested by the increase in cell viability and decrease in pyroptosis rates. Previous studies evidence that *L. pentosus* promotes cognitive capability and alleviates aging-dependent memory impairment [17, 32]. These results dictate the neuron-protective roles of L. pentosus, which is consistent with this study. Therefore, *L. pentosus* may be a promising strategy for neurodegenerative diseases.

BIRC3 plays a vital role in neuronal function. For instance, NPD1-mediated upregulation of BIRC3 promotes neural cell survival [26]. Additionally, cAMP responsive element binding protein interacting with brain derived neurotrophic factor and BIRC3 suppresses A*β*-induced neuronal apoptosis [33]. However, the roles of BIRC3 vary with diseases and cell types. It functions as a protective role in ischemic stroke, Alzheimer's disease, and brain injuries [34] as well as an oncogene [24]. Hence, identifying the roles of BIRC3 in neurodegenerative diseases is of vital importance. In this study, *L. pentosus* alleviated LPS-induced downregulation of BIRC3. However, BIRC3 knockdown alleviated the effects of *L. pentosus* and promoted inflammation and pyroptosis of neurons. These results suggested that BIRC3 may play a neuron-protective role, which is consistent with previous studies [26].

However, approximately 80% studies focused on the roles of BIRC3 cancer. The reports on its roles in neural disorders are limited. BIRC3 mainly exerts its neuron-protective functions via regulating caspases cascades, which suppresses the neuronal apoptosis [26]. Recently, the interplay between pyroptosis and apoptosis has attracted increasing attention. Rogers et al. report that pyroptosis may occur as secondary necrosis after apoptosis [35]. Additionally, pyroptosis and apoptosis may have common signal transduction pathways [36]. In this study, LPS stimulated the activation of NLRC4 inflammasome, which induced cleaved caspase1 and the assembly of N fragments of GSDMD. Additionally, GSDMD-mediated pore formation may orientate neuron to pyroptosis before the onset of apoptosis. However, *L. pentosus*-mediated upregulation of BIRC3 contributed to inactivation of NLRC4 inflammasome, which suppressed neuronal pyroptosis.

In conclusion, *L. pentosus*-induced upregulation of BIRC3 suppressed inflammatory response and pyroptosis of neurons via inactivating NLRC4 inflammasome. Therefore, *L. pentosus* may be an alternative strategy for neurodegenerative diseases.

## Figures and Tables

**Figure 1:** The cell viability of SH-SY5Y cells. The cell viability of SH-SY5Y cells were determined using CCK-8 assay.

**Figure 2:** *L. pentosus* suppressed neuronal inflammatory response. The mRNA levels of IL-18 and IL-1*β* determined using RT-qPCR after treatment with *L. pentosus* for 3, 6, and 12 h. The protein expression of IL-18 and IL-1*β* detected by western blot after treatment with *L. pentosus* for 3, 6, and 12 h. ^*∗*^*P* < 0.05, ^*∗∗*^*P* < 0.01, ^*∗∗*^^*∗*^*P* < 0.001, ^#^*P* < 0.05, ^##^*P* < 0.01, ^###^*P* < 0.001.

**Figure 3:** *L. pentosus* inhibited the pyroptosis of neurons. (a) The cell death of neurons detected using flow cytometry. (b) Neuronal cell death determined using the TUNEL assay. (c) The protein expression of pyroptosis biomarkers, cleaved caspase1, and GSDMD-N detected by western blot. ^*∗∗*^*P* < 0.01, ^##^*P* < 0.01.

**Figure 4:** *L. pentosus* upregulated BIRC3. (a) The mRNA levels of BIRC3 determined using RT-qPCR. (b) The protein expression of BIRC3 detected using western blot. ^*∗∗*^*P* < 0.01, ^##^*P* < 0.01.

**Figure 5:** BIRC3 knockdown promoted inflammatory response and suppressed cell viability of neuronal cells. (a) The mRNA levels of BIRC3 determined using RT-qPCR. (b) The protein expression of BIRC3 detected using western blot. (c) The cell viability of neuronal cells detected using CCK-8. (d) The mRNA levels of IL-18 and IL-1*β* determined using RT-qPCR. (e) The mRNA levels of IL-18 and IL-1*β* detected by western blot. ^*∗∗*^*P* < 0.01, ^##^*P* < 0.01, ^&&^*P* < 0.01.

**Figure 6:** BIRC3 knockdown promoted the pyroptosis of neuronal cells. (a) The cell death of neurons detected using flow cytometry. (b) Neuronal cell death determined using the TUNEL assay. (c) The protein expression of pyroptosis biomarkers, cleaved caspase1, and GSDMD-N detected by western blot. ^*∗∗*^*P* < 0.01, ^##^*P* < 0.01, ^&&^*P* < 0.01.

**Figure 7:** BIRC3 induced the inactivation of NLRC4 inflammasome. (a) The interaction between BIRC3 and inflammasome predicted by STING. (b) The protein expression of NLRP3, NLRP4, NLRP1, and NLRC4.

## Data Availability

The data used to support the findings of this study are included within the article.
